# MSN@IL-4 Sustainingly Mediates Macrophagocyte M2 Polarization and Relieves Osteoblast Damage via NF-*κ*B Pathway-Associated Apoptosis

**DOI:** 10.1155/2022/2898729

**Published:** 2022-10-03

**Authors:** Cheng Shi, Fei Yuan, Zhilong Li, Zhenhua Zheng, Changliang Yuan, Ziyang Huang, Jianping Liu, Xuping Lin, Taoyi Cai, Guofeng Huang, Zhenqi Ding

**Affiliations:** ^1^Department of Orthopedics, Dongnan Hospital of Xiamen University, 269 Zhanghua Middle Road, Zhangzhou, 363000 Fujian, China; ^2^School of Medicine, Xiamen University, 4221 Xiang'an South Road, Xiamen, 361102 Fujian, China

## Abstract

**Background:**

The microenvironment of bone defects displayed that M2 polarization of macrophagocyte could promote the osteoblast growth and benefit the wound healing. Bone scaffold transplantation is considered to be one of the most promising methods for repairing bone defects. The present research was aimed at constructing a kind of novel bone scaffold nanomaterial of MSN@IL-4 for treating bone defects responding to the wound microenvironment of bone defects and elucidating the mechanics of MSN@IL-4 treating bone defect via controlling release of IL-4, inducing M2 polarization and active factor release of macrophagocyte, and eventually relieving osteoblast injury.

**Methods:**

MSN@IL-4 was firstly fabricated and its release of IL-4 was assessed in vitro. Following, the effects of MSN@IL-4 nanocomplex on the release of active factors of macrophage were examined using Elisa assay and promoting M2 polarization of the macrophage by immunofluorescence staining. And then, the effects of active factors from macrophage supernatant induced by MSN@IL-4 on osteoblast growth were examined by CCK-8, flow cytometry, and western blot assay.

**Results:**

The release curve of IL-4 in vitro displayed that there was more than 80% release ratio for 30th day with a sustained manner in pH 5.5. Elisa assay data showed that MSN@IL-4 nanocomplex could constantly promote the release of proproliferative cytokine IL-10, SDF-1*α*, and BMP-2 in macrophagocyte compared to only IL-4 treatment, and immunofluorescent image showed that MSN@IL-4 could promote M2 polarization of macrophagocytes via inducing CD206 expression and suppressing CD86 expression. Osteoblast injury data showed that the supernatant from macrophagocyte treated by MSN@IL-4 could promote the osteoblast proliferation by MTT assay. Flow cytometry data showed that the supernatant from macrophagocyte treated by MSN@IL-4 could suppress the osteoblast apoptosis from 22.1% to 14.6%, and apoptosis-related protein expression data showed that the supernatant from macrophagocyte treated by MSN@IL-4 could suppress the expression of Bax, cleaved caspase 3, and cleaved caspase 8. Furthermore, the immunofluorescent image showed that the supernatant from macrophagocyte treated by MSN@IL-4 could inhibit nucleus location of p65, and western blot data showed that the supernatant from macrophagocyte treated by MSN@IL-4 could suppress the phosphorylation of IKK and induce the expression of I*κ*B.

**Conclusion:**

MSN@IL-4 could control the sustaining release of IL-4, and it exerts the protective effect on osteoblast injury via inducing M2 polarization and proproliferative cytokine of macrophagocyte and following inhibiting the apoptosis and NF-*κ*B pathway-associated inflammation of osteoblast.

## 1. Introduction

Bone defect is a kind of bone deficiency caused by trauma or surgery, which often causes bone nonunion, delayed healing or nonunion, and even local dysfunction [1, 2]. Tissue engineering bone transplantation, mainly composed of bone scaffold materials, seed cells, and cytokines, is considered to be one of the most promising methods for repairing bone defects [3–6]. Although great progress has been made in the research of bone scaffold materials in the past 30 years, its clinical application has not made a breakthrough. The key reason is that the vascularization and osteogenic replacement of tissue-engineered bone scaffolds are slow after transplantation. Some researchers have improved the acceleration of bone regeneration by subcutaneous prevascularization of stents and achieved good results, but this is not feasible in clinical practice [6]. Our previous researches have constructed a series of deproteinized scaffolds which have played a role in the treatment of bone defects to some extent. However, there are still problems such as slow bone growth and poor sustainability. If the microenvironment on the surface of this bone scaffold can be adjusted to make it composite with other bioactive materials to reasonably promote osteogenesis, it will be more ideal and easier to be used in clinic. Therefore, we propose that modifying surface properties of bone scaffolds with bioactive materials may be a potential strategy to improve the healing efficiency of bone defects.

Bone immune response is a common inflammatory process response to bone defect, which runs through the whole process of bone healing and osteoblast growth [7–9]. Macrophages are an important immune regulatory cell of bone immune inflammatory response playing an essential role in phagocytosis of necrotic tissue, detection of bacterial products, and antigen presentation. Macrophages widely exist in periosteum and bone, affecting the maintenance of normal bone morphology and the process of fracture repair. It also exists and acts on multiple stages of fracture repair, producing prosynthetic growth factors at the fracture site and promoting more stable callus formation [10–13]. Macrophages possess many subtypes, and different subtypes can carry out different functions via the polarization transformation according to the changes of the cell environment. In acute inflammatory reaction, macrophages were stimulated by interleukin-2 (IL-2) or liposomes to polarize into M1 type (cd11c+ and ccr7+), which enhanced Th1 helper cells and promoted inflammatory reaction; when stimulated by IL-4, macrophages can polarize into M2 type (cd163+ and cd206+), enhance Th2 helper cell function, reduce inflammation, and promote tissue repair [14, 15].

It has been reported that macrophages cultured on the modified bone scaffold can induce M2 polarization, produce many active bone factors, induce osteoblast proliferation, and eventually promote fracture healing [16]. Although macrophages indirectly participate in the process of bone regeneration, it promotes bone formation by inducing BMP-2 secretion. Many inflammatory cytokines such as IL-4 cannot also directly affect bone metabolism but promote osteoblast growth by inducing macrophage polarization. IL-4-modified tissue engineering bone scaffolds can effectively promote the polarization of macrophages in bone defects and the growth of osteoblasts to achieve the therapeutic effect of bone defects. However, IL-4-modified tissue engineering bone scaffold material still has the problem of one-time release of IL-4, which is difficult to continue to treat bone defects. Therefore, it is necessary to develop tissue engineering bone scaffolds that can control the slow and sustained release of IL-4.

Recently, drug-loaded nanoparticles with controlled release and regulation functions have been widely concerned in the research and development of targeted drugs for various diseases because of their good size and biocompatibility, which can effectively load drug molecules, change their biological distribution and drug metabolism, and control drug release. Among them, the mesoporous silicon nanocarrier (MSN) is a hollow spherical structure with thorns and holes on the surface, which has the characteristics of high specific surface area, good biocompatibility, easy modification, and so on. It is an ideal carrier material for disease treatment drugs. After modification, MSN nanoparticles that respond to low pH, redox reaction, photo enzyme, and other stimuli to control the release of drugs have been reported for many times. MSN nanomaterials can effectively adhere to the surface of deproteinized cancellous bone scaffolds because of their good spines on the surface. Meanwhile, a large number of hydroxyl groups exist on the surface of MSN nanomaterials and can be coupled with IL-4 to form MSN@IL-4 nanocomposites. In a slightly acidic environment, the nanocomposites can slowly release IL-4, so as to achieve the function of sustainable release of IL-4. Therefore, bone scaffold@MSN@IL-4 nanomaterials will be a potentially effective treatment for bone defects.

The present research was aimed at constructing a nanomaterial of bone scaffold@MSN@IL-4 and elucidating its mechanism of promoting fracture healing via the sustaining release of IL-4 to induce M2 polarization of the macrophage to produce many active bone factors causing osteoblast growth. Firstly, the MSN@IL-4 nanocomplex was fabricated and its release of IL-4 was assessed in vitro. Following, the effects of MSN@IL-4 nanocomplex on the release of active factors of macrophage were examined using Elisa assay and promoting M2 polarization of the macrophage by immunofluorescence staining. And then, the effects of active factors from macrophage supernatant induced by MSN@IL-4 on osteoblast growth were examined by CCK-8, flow cytometry, and western blot assay. Bone defect is a kind of bone deficiency caused by trauma or surgery, which often causes bone nonunion, delayed healing or nonunion, and even local dysfunction. Tissue engineering bone transplantation, mainly composed of bone scaffold materials, seed cells, and cytokines, is considered to be one of the most promising methods for repairing bone defects. Although great progress has been made in the research of bone scaffold materials in the past 30 years, its clinical application has not made a breakthrough. The key reason is that the vascularization and osteogenic replacement of tissue-engineered bone scaffolds are slow after transplantation. Some researchers have improved the acceleration of bone regeneration by subcutaneous prevascularization of stents and achieved good results, but this is not feasible in clinical practice. Our previous researches have constructed a series of deproteinized scaffolds which have played a role in the treatment of bone defects to some extent. However, there are still problems such as slow bone growth and poor sustainability. If the microenvironment on the surface of this bone scaffold can be adjusted to make it composite with other bioactive materials to reasonably promote osteogenesis, it will be more ideal and easier to be used in clinic. Therefore, we propose that modifying surface properties of bone scaffolds with bioactive materials may be a potential strategy to improve the healing efficiency of bone defects.

## 2. Methods and Materials

### 2.1. Synthesis of MSN

5 g cetyltrimethylammonium bromide (CTAB, Sigma, USA) was weighted and added into 100 mL of ultrapure water and stirred vigorously for 30 minutes at 90°C until CTAB was completely dissolved. 10 g triethanolamine (TTA, sigma, USA) was weighted and added into 30 mL of ultrapure water to obtain 0.3 mg/mL TTA solution. After that, 5 mL of TTA solution and an additional mixture solution of 30 mL cyclohexane (Sinopharm, China) and 8 mL ethyl orthosilicate (TEOS, Sinopharm, China) were added into the dissolved CTAB solution. The mixed solution reacted under the condition of the continuous stirring at 300 rpm and 90°C for 24 hours. After the reaction, the product of MSN was centrifuged at 1200 rpm for 20 minutes and washed with ethanol and sodium chloride solution for removing the excess raw materials of CTAB. Finally, the prepared MSN was incubated with IL-4 solution, and the product was characterized by scanning electron microscope (SEM).

### 2.2. Elisa Assay for Detecting the Controlled Release of IL-4 from MSN@lL-4

The 100 mg MSN@IL-4 were, respectively, added into the indicated pH (pH 5.5, pH 7.2, and pH 8.8) of phosphate buffer. The buffer was stirred twice per day for 30 days, and the solution was collected at 10 time points of 3^rd^, 6^th^, 9^th^, 12^th^, 15^th^, 18^th^, 21^st^, 24^th^, 27^th^, and 30^th^ day. After that, the collected buffer and the standard substrate were added into the coated wells from Elisa assay kit (R&D, USA) according to the instructions, and the coated plate was shocked and detected for OD value using microplate reader (Thermo, USA). The standard curve of IL-4 was drawn. The contents of IL-4 in buffer were calculated according to the standard curve, and the cumulative release curve of IL-4 was drawn.

### 2.3. Elisa Assay for Detecting the Secretion of Cytokines from Macrophagocyte

The macrophage Raw 264.7 cells (ATCC, USA) were seeded into 12-well plate and cultured for 12 hours. And then, the seeded cells were treated with MSN@IL-4 or MSN for the specific time, and the cell supernatant was collected. After that, the collected supernatant and the standard substrate were added into the coated wells from Elisa assay kit (R&D, USA) according to the instructions, and the coated plate was shocked and detected for OD value using microplate reader (Thermo, USA). The standard curve of IL-10, SDF-1*α*, and BMP-2 was drawn, and their contents in cellular supernatant were calculated.

### 2.4. Immunofluorescent Assay for Detecting the Type of Macrophagocytes

The macrophage Raw 264.7 cells (ATCC, USA) were seeded to the slices in a 24-well plate and cultured for 12 hours. And then, the seeded cells were treated with MSN@IL-4 or MSN for the specific time. After treating, the slices were fixed with 4% formaldehyde (Sinopharm, China) at room temperature for 30 minutes, perforated with 1% triton X-100 solution (Solarbio, China) for 1 hour, blocked with 5% BSA (Aladdin, China) for 1 hour, incubated with primary antibody of CD206 (Abcam, USA) and CD86 (Abcam, USA) for 2 hours, following incubated with the rabbit secondary antibody (Lulong, China) at room temperature, and stained with DAPI (Solarbio, China) and sealed. At last, the slices were imaged by confocal microscope (Carl Zeiss AG, Germany).

### 2.5. MTT Assay for Detecting the Proliferation of Osteoblast

The osteoblast cells were prepared from shin bone of mice and cultured in DMEM medium containing 10% fetal calf serum (FBS, Gibco, USA) for 3 days. And then, the cells were seeded into 96-well plate, cultured in incubator (ThermoFisher, USA) with 5% CO_2_ for 12 hours, and treated with H_2_O_2_ and the secretion supernatant from macrophagocyte subjected to MSN@IL-4. After treating, the cells in wells were added with 20 *μ*L MTT solution (Bio-Tek, China) with the final concentration of 0.5 mg/mL and incubated at 37°C for 2 hours. The precipitate of formazan in the incubated wells of 96-well plates was diluted with 100 *μ*L DMSO (Sigma, USA) per well, and the absorbance at 490 nm was tested by microplate reader (ThermoFisher, USA). The proliferation ratio was calculated as

(1) $$\begin{array}{c} \text{Proliferation rate}=\frac{{\text{OD}}_{\text{sample}}-{\text{OD}}_{\text{blank}}}{{\text{OD}}_{\text{control}}-{\text{OD}}_{\text{blank}}}\times 100\%. \end{array}$$

### 2.6. Flow Cytometry of Dual Staining of FITC-Annexin V/PI for Detecting the Cellular Apoptosis in Osteoblast

The prepared osteoblast cells treated by H_2_O_2_ and the secretion supernatant from macrophagocyte subjected to MSN@IL-4 were digested into single cells with 0.25% trypsin (Biosharp, China) and, following stopping the digestion with DMEM medium with FBS, washed and resuspended with PBS. The resuspended cells were stained via adding 5 *μ*L Annexin V-FITC and PI to incubate at 25°C for 15 minutes according to the instruction from manufacturer (RD, Germany). Finally, the stained osteoblast was diluted with PBS to 1.0 mL and tested using the flow cytometry (BD, USA).

### 2.7. Western Blotting for Detecting the Apoptosis-Related Protein Expression in Osteoblast

The osteoblast cells treated by H_2_O_2_ and the secretion supernatant from macrophagocyte subjected to MSN@IL-4 were collected and lysed with RIPA buffer, and the total protein was harvested and denatured. The denatured proteins were separated by SDS-PAGE and transferred to PVDF membrane (Millipore, USA). The PVDF membrane loading with the protein was blocked with 5% skim milk and incubated with the primary antibodies against Bcl-2 (CST, USA), Bax (CST, USA), caspase 3 (CST, USA), caspase 8 (Abcam, UK), and *β*-actin (CST, USA) at 4°C overnight, following the corresponding secondary antibody (CST, USA). Finally, the band from PVDF membrane was detected by enhanced chemiluminescence solution (ECL, Sigma, USA) and photographic film (Keda, USA).

### 2.8. Immunofluorescent Assay for Detecting the NF-*κ*B Pathway-Related p65 Nuclear Location in Osteoblast

The prepared osteoblast cells were seeded to the slices in a 24-well plate and cultured for 12 hours. And then, the seeded cells were treated with H_2_O_2_ and the secretion supernatant from macrophagocyte subjected to MSN@IL-4 for the specific time. After treating, the slices were fixed with 4% formaldehyde (Sinopharm, China) at room temperature for 30 minutes, perforated with 1% triton X-100 solution (Solarbio, China) for 1 hour, blocked with 5% BSA (Aladdin, China) for 1 hour, incubated with primary antibody of CD206 (Abcam, USA) and CD86 (Abcam, USA) for 2 hours, following incubated with the rabbit secondary antibody (CST, USA) at room temperature, and stained with DAPI (Solarbio, China) and sealed. Finally, the slices were imaged by confocal microscope (Carl Zeiss AG, Germany).

### 2.9. Western Blotting for Detecting the NF-*κ*B Pathway-Related Protein Expression in Osteoblast

The osteoblast cells treated by H_2_O_2_ and the secretion supernatant from macrophagocyte subjected to MSN@IL-4 were collected and lysed with RIPA buffer, and the total protein was harvested and denatured. The denatured proteins were separated by SDS-PAGE and transferred to PVDF membrane (Millipore, USA). The PVDF membrane loading with the protein was blocked with 5% skim milk and incubated with the primary antibodies against p-IKK (CST, USA), IKK (CST, USA), I*κ*B (CST, USA), and *β*-actin (CST, USA) at 4°C overnight, following the corresponding secondary antibody (CST, USA). Finally, the band from PVDF membrane was detected by enhanced chemiluminescence solution (ECL, Sigma, USA) and photographic film (Keda, USA).

### 2.10. Statistical Analysis

By using the software of SPSS and GraphPad, all of the experimental data were presented as themean ± standard deviation(S.D.). The statistical differences among the groups were compared using one-way ANOVA by SPSS of version 19.0 (SPSS, USA). *p* < 0.05 was considered to be statistically significant. The asterisk (∗) represented the comparison with the normal group, and the pound sign (#) was for the comparison with model group.

## 3. Results

### 3.1. Characteristics of MSN@IL-4 Scaffold and IL-4 Release Rate In Vitro

In order to obtain the controlled-release IL-4 system, MSN@IL-4 nanomaterial was fabricated via two-phase process, and in vitro IL-4 release response to pH was evaluated via Elisa assay. SEM photograph of MSN@IL-4 nanoparticle in Figure 1(a) showed that several black spherical particles adhere to the surface of the grey balls, demonstrating that IL-4 was conjugated to MSN. The release curve of IL-4 in vitro (Figure 1(b)) showed that there are 12% release rate for 3^th^ day and more than 80% for 30^th^ day with a sustained manner in pH 5.5, and the release is adequate during 30 days; however, the release rate is only 51% in pH 7.2 and lower than 20% in pH 8.8 for 30^th^ day; even from 15^th^ day, the release is extremely slow or standstill. These release data demonstrate that MSN@IL-4 nanosystem possesses the sustained and adequate IL-4 release potential response to the acid environment.

### 3.2. MSN@IL-4 Promote the Sustaining Secretion of Cytokines of IL-10, SDF-1*α*, and BMP-2 in Macrophagocyte

In order to confirm the effect of fabricated MSN@IL-4 nanomaterial on controlling pro-proliferative cytokine release, the secretion difference of IL-10, SDF-1*α* and BMP-2 in acrophagocyte subjecting to MSN@IL-4 nanocomplex or only IL-4 were detected by Elisa assay. The content curve in Figure 2(a) showed that the cells subjected to MSN@IL-4 nanocomplex treatment with the indicated time displayed a constantly linear increase of IL-10 secretion from 12 hours to 72 hours; however, the content of IL-10 in macrophagocyte subjected to only IL-4 displayed a rising for 24 hours compared to 12 hours and a constant decreasing from 24 hours to 72 hours. The change trends of SDF-1*α* secretion (Figure 2(b)) and BMP-2 secretion (Figure 2(c)) were similar in macrophagocyte subjected to MSN@IL-4 nanocomplex and only IL-4, which were that MSN@IL-4 promotes the constant and time-dependent increase of cytokines and only IL-4 was unsustainable. These results demonstrated that MSN@IL-4 nanocomplex could constantly promote proproliferative cytokine release in macrophagocyte compared to only IL-4 treatment.

### 3.3. MSN@IL-4 Promotes M2 Polarization in Macrophagocyte

To evaluate the promotive effect of MSN@IL-4 on M2 polarization, the M1/M2 indicator of CD86 and CD206 was detected via immunofluorescent experiments. The fluorescent images in Figure 3 showed that macrophagocyte in MSN@IL-4 group displayed a decrease of CD86 expression compared to that in control group (0.01 < ∗*p* < 0.05); oppositely, CD206 expression displayed an increasing trend in cells subjected to MSN@IL-4 nanomaterial compared to that in the control group (0.001 < ∗∗*p* < 0.01). Meanwhile, the cells in only MSN group displayed similar expressions of CD86 and CD206 with that in the control group. These results demonstrated that MSN@IL-4 nanocomplex could promote the M2 polarization of macrophagocyte, but only MSN has no the similar effect.

### 3.4. The Secretion Supernatant from Macrophagocyte Subjected to MSN@IL-4 Protects the Damaged Osteoblast

To confirm the protective effect of M2-polarizationed macrophagocyte on osteoblast, the secretion supernatant from macrophagocyte subjected to MSN@IL-4 was employed to treat the damaged osteoblast, the proliferation was examined via CCK-8 assay and apoptosis was evaluated by flow cytometer. CCK-8 data in Figure 4(a) showed that osteoblast subjected to H_2_O_2_ displayed a decrease of proliferation rate from 100% to 54.7% relative to cells in normal group (0.001 < ∗∗*p* < 0.01), and the osteoblast treated with H_2_O_2_ and the supernatant from macrophagocyte subjected to MSN@IL-4 displayed a reverse enhancement of proliferation rate from 54.7% to 84.2% compared to that in the model group (0.01 < #*p* < 0.05). The scatter diagram of flow cytometer in Figure 4(b) showed that osteoblast subjected to H_2_O_2_ displayed an increase of apoptosis rate from 7.5% to 27.3% relative to cells in the normal group (0.001 < ∗∗*p* < 0.01), and the osteoblast treated with H_2_O_2_ and the supernatant from macrophagocyte subjected to MSN@IL-4 displayed a reverse decrease of apoptosis rate from 27.3% to 14.5% compared to that in the model group (0.01 < #*p* < 0.05). These results demonstrated that the supernatant from the M2-polarizationed macrophagocyte induced by MSN@IL-4 could protect the osteoblast from H_2_O_2_-induced injury.

### 3.5. The Secretion Supernatant from Macrophagocyte Subjected to MSN@IL-4 Suppresses the Apoptosis-Related Protein Expression in Osteoblast

To further confirm the protective effect of M2-polarizationed macrophagocyte on the apoptosis during osteoblast injury, the apoptosis-associated proteins of bcl-2, bax, caspase 3, and caspase 9 were probed using western blotting. The band images in Figure 5 showed that osteoblast subjected to H_2_O_2_ displayed the expression increase of bax (∗∗*p* < 0.01), cleaved caspase 3 (∗∗*p* < 0.01), and cleaved caspase 8 (∗∗*p* < 0.01) relative to cells in the normal group. Expectantly, the osteoblast treated with H_2_O_2_ and the supernatant from macrophagocyte subjected to MSN@IL-4 displayed a reverse regulation of protein expression that bax (##*p* < 0.01), cleaved caspase 3 (#*p* < 0.05), and cleaved caspase 8 (#*p* < 0.05) were inhibited relative to cells in the model group. These results were consist with the apoptosis data from flow cytometry, demonstrating that the supernatant from the M2-polarizationed macrophagocyte induced by MSN@IL-4 could protect the osteoblast from H_2_O_2_-induced apoptosis.

### 3.6. The Secretion Supernatant from Macrophagocyte Subjected to MSN@IL-4 Suppresses the NF-*κ*B Pathway-Related p65 Nuclear Location in Osteoblast

To evaluate the inhibitory effect of M2-polarizationed macrophagocyte on osteoblast inflammation, p65 nucleus location, a classical NF-*κ*B pathway indicator, was probed via immunofluorescent experiments. The fluorescent images in Figure 6 showed the osteoblast treated with H_2_O_2_ and the supernatant from macrophagocyte subjected to MSN@IL-4 displayed a inhibitory effect of p65 nucleus location compared that in the model group and have the significant statistical difference of 0.01 < ∗∗*p* < 0.01; however, the osteoblast treated with H_2_O_2_ and the supernatant from macrophagocyte subjected to MSN displayed a weak inhibitory of p65 nucleus location with no statistical difference compared that in the model group. The result demonstrated that the supernatant from the M2-polarizationed macrophagocyte induced by MSN@IL-4 could suppress the osteoblast inflammation via NF-*κ*B p65 nuclear location.

### 3.7. The Secretion Supernatant from Macrophagocyte Subjected to MSN@IL-4 Suppresses the NF-*κ*B Pathway-Related Protein Expression in Osteoblast

To further confirm the suppressive effect of M2-polarizationed macrophagocyte on inflammation during osteoblast injury, the NF-*κ*B pathway-associated proteins of p-IKK, IKK, and I*κ*B were probed using western blotting. The band images in Figure 7 showed that osteoblast subjected to H_2_O_2_ displayed a evident decrease of I*κ*B expression (∗∗*p* < 0.01) and the phosphorylation increase of IKK (∗∗*p* < 0.01) relative to cells in the normal group. Expectantly, the osteoblast treated with H_2_O_2_ and the supernatant from macrophagocyte subjected to MSN@IL-4 displayed a reverse regulation of protein expression that I*κ*B expression in osteoblast cells of MSN@IL-4 group was induced (##*p* < 0.01) and the protein phosphorylation of IKK was inhibited (#*p* < 0.05) relative to cells in the model group. These results were consistent with the p65 nuclear location from immunofluorescent, demonstrating that the supernatant from the M2-polarizationed macrophagocyte induced by MSN@IL-4 could suppress NF-*κ*B pathway-associated inflammation in osteoblast.

## 4. Discussion

It is commonly recognized that a large number of inflammatory cells infiltrated at the injury site of bone defect, and inflammatory cells under different conditions will have different subtypes exerting diametrically opposite regulatory effects on osteoblasts of wound [17–19]. M2-polarized macrophages can play an importantly role in wound healing by promoting the secretion of proosteocyte growth factors [20, 21]. Therefore, the supplement of inducer of macrophage-M2-polarizaition such as IL-4 into the wound of bone defect would effectively promote wound healing. At present, the main treatment method for bone defects is bone transplantation. We have also reported the therapeutic effect of deproteinized bone scaffolds in the treatment of bone defects. However, the modified bone scaffolds added with macrophage M2 polarization inducers such as IL-4 have rarely been reported in the treatment of bone defects. Meanwhile, how to control the release of IL-4 in the modified bone scaffold to achieve sustained induction of macrophage polarization is also a technical problem. In this project, we constructed a nanomaterial of MSN@IL-4 loaded on a deproteinized bone scaffold, which can continuously and slowly release IL-4 in response to a slightly acidic environment. We found that MSN@IL-4 could promote the sustaining secretion of cytokines of IL-10, SDF-1*α*, and BMP-2 compared to only IL-4 and induced M2 polarization in macrophagocyte. The supernatant from macrophagocyte treated with MSN@IL-4 was added into the damaged osteoblast by H_2_O_2_, the proliferation ratio of the damaged osteoblast increased, the apoptosis ratio decreased, and NF-*κ*B-associated inflammation was inhibited. These results demonstrated that MSN@IL-4 could protect osteoblast against cell injury induced H_2_O_2_ via macrophagocyte M2 polarization and sustainingly promoted the release of active osteoblast factor.

Apoptosis is considered as a physiologically and pathologically programmed cell death process to clear off the redundant and malfunctional cells for keeping the cellular homeostasis [22]. Mitochondrial exerts the roles of the controlling center for cellular activities, which masters the oxidative phosphorylation and respiratory chain regulating almost all of the cellular physiopathology including apoptosis. During the apoptosis progression, apoptosis stimuli initiate the mitochondrial depolarization, induces/inhibits the expression of apoptosis-associated proteins of bax, bad, and bcl-2 from mitochondrial, triggers the cysteinyl aspartate specific proteinase (caspase) of caspase 3, caspase 8, and caspase 9, and consequently activates the cleavage of poly ADP-ribose polymerase (PARP), cell death, and tissue damage [23]. In the present research, H_2_O_2_ initiate the osteoblast apoptosis via regulating bax and bcl-2 expression and evoking caspase activities. Oppositely, the supernatant from macrophagocyte treated by MSN@IL-4 relieved the apoptosis induced by H_2_O_2_. These data demonstrated that MSN@IL-4 could relieve osteoblast injury via inducing macrophagocyte release the active cellular factors.

The nuclear factor *κ*B pathway (NF-*κ*B pathway) has long been considered as a prototypical proinflammatory signaling pathway and controlled the expression of proinflammatory genes including cytokines, chemokines, and adhesion molecules [24]. NF-*κ*B pathway was initiatively trigged with the phosphorylation of IKK response to inflammation factor, following the phosphorylation and degradation of I*κ*B and then release the p65 protein from the complex of p65/p115/I*κ*B, and induced its translocation from cytoplasm to nucleus for activating the gene expression of inflammatory factor such as TNF*α*, IL-1*β*, and IL-6, consequently causing the development of chronic diseases including cancer, diabetes, and osteoarthritis. In the present research, we found that the osteoblast damaged by H_2_O_2_ displayed an obvious phosphorylation of IKK, degradation of I*κ*B, and phosphorylation of p65; meanwhile, the cells treated with the supernatant from macrophagocyte treated by MSN@IL-4 had a reverse trend change of the above NF-*κ*B pathway indicators, demonstrating that MSN@IL-4 could protect against H_2_O_2_-inducing osteoblast injury via the induction of macrophagocyte release of the active cellular factors inhibiting the NF-*κ*B inflammation pathway in osteoblast (Figure 8).

## Figures and Tables

**Figure 1:** The scaffold of MSN@IL-4 and IL-4 release from MSN@IL-4 in vitro. (a) SEM image of MSN@IL-4 and (b) cumulative release of IL-4 response to pH.

**Figure 2:** The effect of MSN@IL-4 nanomaterials for promoting the sustaining secretion of cytokines of IL-10, SDF-1*α*, and BMP-2 in macrophagocyte. Elisa assay for detecting the contents of IL-10 (a), SDF-1*α* (b), and BMP-2 (c) in the cellular supernatant.

**Figure 3:** The promotive effect of MSN@IL-4 nanomaterials on M2 polarization in macrophagocyte. The representative fluorescent images of the stained CD86 and CD206 were displayed and relative expression were analyzed using GraphPad software. ∗*p* < 0.05 and ∗∗*p* < 0.01 vs. control group.

**Figure 4:** The protective effect of the secretion supernatant from macrophagocyte subjected to MSN@IL-4 nanomaterial against H_2_O_2_-induced osteoblast injury. (a) CCK-8 assay for detecting the cellular proliferation of the normal osteoblast (normal group), H_2_O_2_-treated osteoblast (model group), and the treated osteoblast with H_2_O_2_ and supernatant from macrophagocyte subjected to MSN@IL-4 nanomaterial (MSN@IL-4 group). (b) Flow cytometry analysis with dual staining of PI and FITC-annexin V for testing the cellular apoptosis rate. (c) The statistical analysis for the apoptosis rate using GraphPad software. ∗∗*p* < 0.01 and ∗∗∗*p* < 0.001 vs. normal group; #*p* < 0.05 vs. model group.

**Figure 5:** The regulatory effect of the secretion supernatant from macrophagocyte subjected to MSN@IL-4 nanomaterial on apoptosis-associated proteins of bcl-2, bax, cleaved caspase 3, and cleaved caspase 8. ∗∗*p* < 0.01 vs. normal group; #*p* < 0.05 and ##*p* < 0.01 vs. model group.

**Figure 6:** The inhibitive effect of the secretion supernatant from macrophagocyte subjected to MSN@IL-4 nanomaterial on the NF-*κ*B pathway. The nucleus location of p65 in H_2_O_2_-treated osteoblast (model group) and the treated osteoblast with supernatant from macrophagocyte subjected to MSN@IL-4 nanomaterial (MSN@IL-4 group) or only MSN (MSN group). The statistical analysis of p65 nucleus location using GraphPad software. ∗∗*p* < 0.01 vs. model group.

**Figure 7:** The regulatory effect of the secretion supernatant from macrophagocyte subjected to MSN@IL-4 nanomaterial on NF-*κ*B pathway-associated proteins of p-IKK, IKK, and I*κ*B. ∗*p* < 0.01 vs. normal group; #*p* < 0.05 and ##*p* < 0.01 vs. model group.

**Figure 8:** Scheme summarizing MSN@IL-4 relieving osteoblast damage via macrophagocyte M2 polarization.

## Data Availability

The data supporting the findings of this article will be available by the authors.
